The article "Scutellarein inhibits cancer cell metastasis in vitro and attenuates the development of fibrosarcoma in vivo" was published in 2014. Journal: Int J Mol Med.

# Scutellarein inhibits cancer cell metastasis *in vitro* and attenuates the development of fibrosarcoma *in vivo*

**DOI:** 10.3892/ijmm.2014.1997

**Published:** 2014-11-12

**Authors:** XIUJUAN SHI, GUANGFENG CHEN, XIAOQIANG LIU, YU QIU, SHUZHANG YANG, YAN ZHANG, XUEXUN FANG, CHEN ZHANG, XIAOQING LIU

**Affiliations:** 1 Tenth People’s Hospital, Tongji University School of Medicine, Shanghai 200072, P.R. China; 2 Key Laboratory for Molecular Enzymology and Engineering of the Ministry of Education, Jilin University, Changchun, Jilin 130023, P.R. China

**Keywords:** scutellarein, HT1080 cells, matrix metalloproteinase, metastasis, invasion

## Abstract

Fibrosarcoma is an aggressive and highly metastatic cancer of the connective tissue, for which effective therapeutic methods are limited. Recently, there has been a renewed interest in small molecular compounds from natural products in the treatment of cancer. In the present study, we investigated the compound, scutellarein, extracted from the perennial herb *Scutellaria lateriflora*, and it was found to possess anticancer potential. Cell proliferation assay and cell cycle analysis revealed that the proliferation rate of HT1080 human fibrosarcoma cells was significantly suppressed by treatment with scutellarein through the induction of apoptosis. Moreover, an *in vivo* experiment using Balb/c nude mice revealed that the volume and weight of the tumors were markedly reduced following treatment with scutellarein. We also analyzed the effects of scutellarein on the markers of metastasis, using the HT1080 cells. The results indicated that scutellarein potently inhibited cell migration, invasion and the expression and activity of matrix metalloproteinase (MMP)-2, -9 and -14. Furthermore, MMP activation and cell survival were suppressed due to the scutellarein-mediated downregulation of nuclear factor κ-light-chain-enhancer of activated B cells (NF-κB) activation. In conclusion, our data suggest that scutellarein has the ability to attenuate the development of fibrosarcoma and inhibit cancer cell metastasis.

## Introduction

Cancer, the leading cause of mortality worldwide, can be defined by 6 hallmarks, including uncontrollable growth, immortality and the ability to invade other tissues (1). The primary tumor eventually transforms into a malignant phenotype through a series of progressive physiological changes. The malignant phenotype leads to the spread of the tumors through metastasis. The invasion and development of a secondary tumor involves a series of sequential steps, such as intravasation into the circulatory system and extravasation to a secondary site (2). Not all tumor cells successfully metastasize to distant sites, forming new tumors. Although metastases cause 90% of human cancer-related deaths, they are not responsible for the development of the primary tumor (10).

Tumor cell dissemination, epithelial-mesenchymal transition (EMT), invasion and cell migration are the initial and critical steps of the metastatic cascade (3,4). EMT results in the secretion of extracellular matrix (ECM) protein-degrading enzymes, which in turn facilitate the invasion and migration of tumor cells by remodeling the ECM within the tumor micro-environment. Extracellular proteinases, such as matrix metalloproteinases (MMPs), initiate the changes required for tumor metastasis, with the degradation of the basement membrane (type IV collagen) playing a key role during invasion and metastasis (5). MMPs and zinc-dependent endopeptidases, members of a large family of proteases, are known to carry out vital functions in normal physiology, including tissue remodeling and organ development (6–8). By contrast, tumor cells overexpress MMPs or dysregulate their activities. Specifically, MMP-1, -2, -3, -7, -9, -13 and -14 actively contribute to tumor progression (9). MMPs not only modify the tumor microenvironment, but also inhibit the apoptosis of cancer cells by cleaving and clearing death receptors, and eventually misguiding the tumor immune surveillance (10). Thus, MMPs have long been a target of cancer chemotherapy. However, various types of MMP inhibitors have failed to increase the survival rate. It is, therefore, important to explore the advanced antitumor functions and underlying mechanisms of action of MMP inhibitors (11).

Scutellarein (5,6,7,4′-tetrahydroxyflavone), a flavone found in the perennial herb, *Scutellaria lateriflora*, has a range of biological activities (12). The high bioavailability of scutellarein has been attributed to its improved solubility compared with scutellarin (40,5,6-trihydroxyflavone-7-glucuronide), which is the most comprehensively studied active ingredient of the herb. In addition, scutellarin is mainly absorbed in the form of its hydrolyzed product, scutellarein, which is more active than scutellarin (13). A previous study demonstrated the significant anticancer activity of scutellarein (the main constituent of *Scutellaria barbata* extract) in human colon cancer cell lines (14). In the present study, we investigated the potential of scutellarein to attenuate the development of fibrosarcoma *in vivo,* as well as and its inhibitory effects on the migration and invasion of HT1080 fibrosarcoma cells *in vitro*.

## Materials and methods

### Drugs

Scutellarein (purity ≥98%) and 3-(4,5-dimethylthiazol-2-yl)-2,5-diphenyltetrazolium-bromide (MTT) were purchased from Sigma-Aldrich Inc. (St. Louis, MO, USA). HT1080 human fibrosarcoma cells were purchased form the American Type Culture Collection (ATCC, Manassas, VA, USA). Dulbecco’s modified Eagle’s medium (DMEM), fetal bovine serum (FBS), penicillin, streptomycin, trypsin, phosphate-buffered saline (PBS) with calcium chloride and magnesium chloride were obtained from Gibco-Life Technologies (Carlsbad, CA, USA). Culture inserts used for wound healing assay were obtained from ibidi GmbH (Munich, Germany). The BD Cycletest Plus DNA reagent kit and Matrigel™ used for the invasion assay were purchased from BD Biosciences (Franklin Lakes, NJ, USA). Primary antibodies for western blot analysis were as follows: rabbit anti-human MMP2 (#sc-10736; Santa Cruz Biotechnology, Santa Cruz, CA, USA), goat anti-human MMP9 (#sc-6840; Santa Cruz Biotechnology), goat anti-human MMP14 (#sc-12367; Santa Cruz Biotechnology), rabbit anti-human pIκB (#2859s; Cell Signaling Technology, Danvers, MA, USA), rabbit anti-human IκB (#10268-1-AP; ProteinTech, Chicago, IL, USA), rabbit anti-human NF-κB (#10745-1-AP; ProteinTech), rabbit anti-human histone-H3 (#17168-1-AP; ProteinTech). Goat anti-rabbit IgG peroxidase conjugate (#a9169; Sigma-Aldrich, and rabbit anti-goat IgG peroxidase conjugate (#a5420; Sigma-Aldrich) were used as secondary antibodies. All other chemicals and reagents used in the study were of analytical grade and commercially available.

### Cell culture

HT1080 human fibrosarcoma cells were maintained in DMEM supplemented with 10% FBS, 100 U/ml streptomycin and 100 U/ml penicillin at 37°C in a humidified incubator containing 5% CO_2_. The cells were used after a minimum of 5 passages and experiments were performed at confluence.

### Cell viability (MTT) assay

The cytotoxic effects of scutellarein towards HT1080 cells were evaluated by MTT assay as previously described in the study by Chen *et al* (15). Briefly, the cells were plated in 48-well plates at a density of 1×10^4^ cells/well and incubated overnight. The cells were then washed with fresh medium and incubated with 200 μl of fresh medium containing 2 different concentrations (10 and 50 μm/l) of scutellarein dissolved in 10% dimethyl sulfoxide (DMSO) for 24 h. DMSO was used as the vehicle control in this experiment. The final concentration of DMSO in the culture medium was <0.1% (v/v). Following incubation, 20 μl of MTT solution (1 mg/ml) were added to each well followed by incubation for a further 4 h at 37°C, after which the MTT solution in each well was aspirated and 100 μl of DMSO were added to dissolve the formazan crystals. The optical density of each well was measured at 490 nm using a microplate reader (Tecan Group Ltd., Grödig, Austria). The cytotoxicity of the compound, scutellarein, was compared with that of the vehicle, DMSO.

### Cancer cell migration assay

The culture inserts, consisting of 2 reservoirs separated by a 500-mm thick wall, were placed in a 24-well plate. An equal amount (70 μl) of HT1080 cell suspension (5×10^5^ cells/ml) was added to each reservoir followed by incubation at 37°C. After the cells attached completely (10 h), the culture inserts were gently removed and the wells were filled with serum-free culture medium containing 0.2% bovine serum albumin (BSA) in the presence or absence of scutellarein. The control of the experiment was set by the addition of DMSO alone. The gap between 2 cell layers was observed under a microscope (IX71; Olympus, Tokyo, Japan) immediately and after 6 h of treatment.

### Colony forming assay

The cells were maintained in DMEM supplemented with 10% FBS, 1% penicillin/streptomycin and 1×10^3^ cells were plated in a 3.5-cm dish followed by incubation at 37°C overnight. Various concentrations of the compound, scutellarein (10 and 50 μm/l), were added to each dish followed by incubation for 15 days. The cells treated with the vehicle alone (DMSO) were maintained as the negative control. After 15 days, each well was washed with 1 ml PBS followed by the addition of 1 ml crystal violet solution (1% crystal violet and 10% ethanol). After 10 min of incubation, the excess crystal violet was washed out with PBS and the stained colonies were counted.

### In vitro invasion assay

The invasion of the HT1080 cells was monitored *in vitro* using BD Matrigel™-coated 24-well Transwell units. Briefly, the Matrigel-coated Transwells were washed thoroughly with PBS and dried before use. The cells (200 μl; 2.5×10^5^ cells/ml of serum-free medium) were added to each filter chamber followed by incubation for 4 h for complete attachment. The cells were subsequently treated with various concentrations of scutellarein. The Transwells were placed into the lower chamber containing 750 μl of serum with DMEM and incubated for 36 h. The medium in the upper chamber was then removed and washed twice with PBS. The cells were fixed by the addition of formaldehyde and permeabilized with 100% methanol. The methanol-permeablilized cells were stained with crystal violet (Sigma-Aldrich). The excess stain was removed by washing twice with PBS. Non-invasive cells on the upper side of the Transwell were scraped off with a cotton swab and cells on the bottom side were observed under a microscope (IX71; Olympus). For quantification, the cells stained with crystal violet were dissolved in acetic acid and absorbance was read at 600 nm using a Bio-Rad 680 microplate reader (Bio-Rad Laboratories, Hercules, CA, USA).

### Cell cycle analysis

The analysis of the cell cycle of HT1080 cells was carried out according to the manufacturer’s instructions (BD Cycletest assay, BD Biosciences). Briefly, the HT1080 cells in the exponential growth phase were seeded in a 6-well plate at a density of 2×10^5^ cells/ml and incubated overnight at 37°C. The culture medium was changed to 10% FBS supplemented with DMEM containing 10 and 50 μm/l of scutellarein or the vehicle (DMSO) followed by 24 h of incubation at 37°C. Following incubation, the cells were harvested into 15-ml tubes and centrifuged (800 rpm, 5 min) at room temperature. The harvested cells were fixed by the addition of 90% methanol, drop-wise to the cell pellet, and the cell suspension was incubated for 30 min at 4°C. A cell pellet was obtained by centrifugation at 800 rpm followed by washing twice with PBS. The pellet was then resuspended in propidium iodide and incubated at 37°C for 1 h. Data were analyzed using a fluorescence-activated cell sorting machine (FACSCalibur flow cytometer; BD Biosciences). The acquired FACS data were analyzed by ModFit LT software (Verity Software House, Inc., Topsham, ME, USA).

### Measurement of MMP-2 and MMP-9 activity by gelatin zymography

The HT1080 cells (2×10^5^ cells/ml) in DMEM containing 10% FBS were seeded in 24-well plates and incubated overnight at 37°C. The following day, the culture medium was changed to serum-free, fresh medium containing 10 and 50 μm/l of scutellarein or vehicle (DMSO), and incubated for 24 h at 37°C. Following incubation, the conditioned medium was collected, and the protein content was determined by Bradford assay. Equal amounts of protein were electrophoresed on 10% SDS-PAGE containing 0.1% gelatin. The electrophoresed gel was then washed with 50 mM Tris-HCl (pH 7.5) containing 2.5% Triton X-100, followed by incubation overnight at 37°C in a developing buffer containing 10 mM CaCl_2_, 50 mM Tris-HCl and 150 mM NaCl. Following incubation, the gel was stained with 0.5% coomassie brilliant blue dye in 30% methanol and 10% acetic acid to visualize the areas of gelatin hydrolyzed by the MMPs. Finally, the bands were observed by removing the stain using water.

### Quantitative reverse transcription-polymerase chain reaction (RT-qPCR)

RT-qPCR was performed to detect the mRNA expression levels of MMP-2, MMP-9 and MMP-14 in the HT1080 cells treated with the compound, scutellarein, and the vehicle according to the manufacturer’s instructions (Invitrogen, Carlsbad, CA, USA). Briefly, the cells were grown in a 60-mm culture dish, treated with scutellarein (10 and 50 μm/l) or the vehicle (DMSO) and incubated for 6 h at 37°C. Total cellular RNA was extracted from the treated cells by lysing the cells with TRIzol reagent (Gibco, Carlsbad, CA, USA) followed by centrifugation at 12,000 rpm for 15 min at 4°C with chloroform (in 5:1 ratio). The supernatant was centrifuged with isopropanol (in 1:1 ratio) at 10,000 rpm for 10 min. The RNA pellet was washed with 75% ethanol and solubilized with diethyl pyrocarbonate (DEPC)-treated water. RNA was quantified by measuring the absorbance at 260 nm using a NanoDrop ND-1000 spectrophotometer (Thermo Fisher Scientific, Waltham, MA, USA). Single-stranded cDNA was prepared using a Reverse Transcription system (Promega, Madison, WI, USA). The mRNA expression of the target gene was determined by SYBR-Green assays. SYBR-Green qPCR SuperMix-UDG was purchased from Invitrogen. Quantitative PCR was performed using an Applied Biosystems 7300 Sequence Detection system. All experiments were performed in triplicate. The relative gene expression levels were calculated using the 2^−ΔΔCT^ analysis tool. The primers used for PCR were as follows: MMP-2 forward, 5′-CTGCGGTTTTCTCGAATCCATG-3′ and reverse, 5′-GTCCTTACCGTCAAAGGGGTATCC-3′; MMP-9 forward, 5′-GAGGCGCTCATGTACCCTATGTAC-3′ and reverse, 5′-GTTCAGGGCGAGGACCATAGAG-3′; MMP-14 forward, 5′-CTTCCGTGGAAACAAGTACTACCGT-3′ and reverse, 5″-ATCCCTTCCCAGACTTTGATGTTC-3″; and β-actin (ACTB; internal control) forward, 5″-CCCTGGCACCCA GCAC-3″ and reverse, 5″-GCCGATCCACACGGAGTAC-3″.

### Western blot analysis

The expression levels of the proteins of interest in the treated HT1080 cells were analyzed using standard western blot analysis. In this procedure, the treated cells were lysed with RIPA buffer (Sigma-Aldrich) on ice for 5 min. The cytosolic and nuclear fractions were separated using the Nuclear/Cytosol fractionation kit (BioVision Technologies, Exton, PA, USA) following the manufacturer’s instructions, where necessary. Cell lysates (20 μg of total proteins) were separated by SDS-PAGE and electroblotted onto nitrocellulose membranes. The membranes were blocked with 5% BSA for 2 h at room temperature and incubated with different antibodies overnight at 4°C. This was followed by incubation with relevant secondary antibodies for 1 h at room temperature. Protein bands were visualized using the Chemiluminescent ECL assay kit (Amersham Pharmacia Biosciences) and an LAS-3000^®^ Luminescent image analyzer. Protein expression levels were quantitatively determined using ImageJ software (National Institutes of Health, Bethesda, MD, USA). β-actin and glyceraldehyde-3-phosphate dehydrogenase (GAPDH) were used as internal references for protein expression in the treated HT1080 cells.

### Animal experiments

The effects of scutellarein on tumor progression were monitored using a nude mouse model. Male Balb/c nude mice (5 weeks old) were purchased form SLAC Laboratory Animal Co. (Shanghai, China), and all mice were maintained according to animal welfare regulations and protocols approved by the Institutional Animal Care and Use Committee of Tongji University (Shanghai, China). The HT1080 cells (1×10^7^ cells/mouse) were injected subcutaneously into the right forelimb axillary region of Balb/c nude mice to generate tumors. After the tumors had grown, the mice were randomly separated into 3 groups and treated with scutellarein (0.05 and 0.5 μg/g) via intraperitoneal injection. The control group in the experiment was treated with the same amount of PBS. The mice were sacrificed by cervical dislocation after 20 days and the tumor weight and volume of each mouse were evaluated.

### Statistical analysis

All the results are representative of 3 or more independent experiments, with the data expressed as the means ± SD. Differences between the control and treatment groups were analyzed using the Student’s t-test with SPSS 17.0 software. A P-value <0.05 was considered to indicate a statistically significant difference.

## Results

### Anti-proliferative effects of scutellarein against HT1080 fibrosarcoma cells

Scutellarein, found in *Scutellaria lateriflora* and other members of the genus *Scutellaria*, is a member of the flavone group of phenolic compounds (Fig. 1A). The viability of the HT1080 fibrosarcoma cells in the presence of scutellarein at various concentrations and the vehicle (DMSO) was assessed with MTT assay. In comparison to the DMSO-treated cells, the cells treated with 10 and 50 μm/l of scutellarein showed a 27.6 and 32.8% reduction in cell viability, respectively (Fig. 1B). The suppressive effects of scutellarein on the viability of the HT1080 fibrosarcoma cells clearly demonstrates its anti-proliferative activity (Fig. 1C).

### Scutellarein inhibits cell colony formation and promotes apoptosis

To further investigate the anti-proliferative effects of scutellarein on human fibrosarcoma, we performed a cell colony formation assay. The plates with scutellarein-treated cells showed few cell clones, whereas the vehicle (DMSO)-treated cell plates presented a clear colony formation of HT1080 cells (Fig. 2A). In addition, the quantification analysis revealed that the average cell clone number of the cells treated with scutellarein at concentrations of 10 and 50 μm/l was 2.6 and 0.2, respectively, while the DMSO treated group displayed a cell clone number of 75 (Fig. 2B). Furthermore, cell apoptosis detection assay was performed to determine whether scutellarein promotes the apoptosis of fibrosarcoma cells. Flow cytometric analysis revealed that the rate of apoptosis following treatment with 10 μm/l scutellarein was 42.16%; this increased to 43.12% following treatment with 50 μm/l scutellarein, while for the DMSO-treated cells, the rate of apoptosis was 5.16%. These results clearly indicate that scutellarein significantly increases the number of apoptotic cells (Fig. 2C).

### Scutellarein attenuates fibrosarcoma in vivo

Based on our results demonstrating that scutellarein inhibited proliferation and promoted apoptosis *in vitro*, we wished to determine whether this compound attenuates the development of fibrosarcoma *in vivo*. Fibrosarcoma formation was induced by injecting HT1080 cells into Balb/c nude mice. At 20 days following the injection of the cancer cells, the tumor-bearing mice were sacrificed by cervical dislocation and the solid tumors were removed and arranged with their weights measured and analyzed (Fig. 3A). The injection of scutellarein at doses of 0.05 and 0.5 μg/g, suppressed the tumor weight by 30.25 and 46.17%, respectively, in comparison to the control group treated with PBS (Fig. 3B). The tumors were also measured using a caliper, and the tumor volume was calculated as the arithmetic mean of 2 perpendicular diameters. Statistical analysis revealed that treatment with scutellarein at a dose of 0.5 μg/g reduced the tumor volume by 47.4% when compared with the PBS-treated control group. Similar results were observed following treatment with a lower concentration (0.05 μg/g) of scutellarein (tumor volume was reduced by 47%; Fig. 3C).

### Scutellarein decreases metastasis in vitro

To evaluate the antimetastatic potential of scutellarein, cell migration assay and invasion assay were performed. The vehicle (DMSO)-treated HT1080 cells migrated towards the empty area after 6 h of incubation. However, the scutellarein-treated cells showed a significant dose-dependent reduction in their migration ability, suggesting that scutellarein reduced the HT1080 cell migration (Fig. 4A). Due to the ability of cells to invade through Matrigel, the effects of scutellarein on the invasion of HT1080 cells were determined by a standardized cell Transwell invasion assay. A plethora of HT1080 cells treated with the vehicle invaded the Matrigel, while the scutellarein-treated cells showed a decrease in cell invasion in a dose-dependent manner (Fig. 4B). Optical absorbance at 600 nm was measured based on crystal violet staining of the cancer cells. Quantification analysis indicated that the highest concentration of scutellarein used, induced a 3-fold decrease in cell invasion (Fig. 4C). Taken together, these observations indicate that scutellarein has the potential to decrease cancer cell metastasis *in vitro*.

### Effect of scutellarein on the expression and activity of MMPs in HT1080 cells

To explore the mechanisms of the scutellarein-mediated inhibition of cell migration, the gene expression levels of cell migration-related proteins, MMP-2, -9 and -14, were analyzed by qRT-PCR. The expression level of human β-actin (ACTB) was used as an internal control. As compared to the vehicle (DMSO)-treated cells, the expression levels of MMP-2, -9 and -14 were significantly reduced following treatment with scutellarein. However, the inhibition efficiency varied among these genes. The inhibition efficiency of scutellarein on the activity of MMP-2 and -9 was dose-dependent. By contrast, the inhibition efficiency of 10 μm/l scutellarein on MMP-14 activity was 67%, while that of 50 μm/l scutellarein was 58%, suggesting a non-dose-dependent pattern (Fig. 5A). The effects of scutellarein on the activity of gelatinases (MMP-2 and -9) was confirmed by performing gelatin zymography, which clearly indicated that scutellarein inhibited both MMP-2 and -9 activity in a dose-dependent manner (Fig. 5B). Western blot analysis, carried out to ascertain the levels of MMP-2, -9 and 14, revealed that MMP-2 and -9 protein expression was suppressed by treatment with scutellarein in a dose-dependent manner, as compared to the vehicle-treated control. This result was in agreement with the results of RT-qPCR. However, in contrast to the RT-qPCR data, the protein level of MMP-14 was inhibited by treatment with scutellarein in a dose-dependent manner (Fig. 5C).

### Scutellarein inhibits the activation of the nuclear factor κ-light-chain-enhancer of activated B cells (NF-κB) signaling pathway

Cell migration and proliferation are controlled by complex cellular signaling pathways. The NF-κB signaling pathway is crucial for migration and cell survival (16,17). The effects of scutellarein on the regulation of the NF-κB signaling pathway were determined by western blot analysis. The NF-κB transcription factor is translocated from the cytosol to the nucleus upon activation. The nuclear NF-κB levels were significantly suppressed following treatment with scutellarein and the inhibition was dose-dependent (Fig. 6A). Quantification analysis revealed that, at the highest concentration of scutellarein, the nuclear NF-κB levels were reduced by up to 5-fold compared to the vehicle (DMSO)-treated cells (Fig. 6B). The cytosolic NF-κB levels also increased in a dose-dependent manner. Furthermore, the cytosolic levels of IκB and p-IκB were analyzed. The results indicated that treatment with scutellarein increased the cytosolic IκB levels in a dose-dependent manner, suppressing IκB phosphorylation. In conclusion, these data suggest that scutellarein regulates the proliferation and migration of HT1080 cells by inhibiting the activation of the NF-κB signaling pathway.

## Discussion

Natural products have been the single most productive source for the development of drugs, particularly as anticancer agents (18,19). Scutellarin, clinically used in the treatment of acute cerebral infarction and paralysis in China, is a natural product extracted from the Chinese herb, *Erigeron breviscapus* (Vant.) Hand-Mazz (20). Previous studies have demonstrated that scutellarin has anticancer properties (21,22). However, the water-solubility and bioavailability of scutellarin is low (23). It has been reported that scutellarein has relatively better solubility, bioavailability and bio-activity compared to scutellarin (13). Based on these observations, the present study was designed to investigate the ability of scutellarein as a lead compound to attenuate the development of human fibrosarcoma by using *in vitro* and *in vivo* models. Our results revealed that scutellarein has the potential to inhibit tumor formation and the metastasis of fibrosarcoma cells.

Metastasis, accounting for over 90% of cancer-related deaths worldwide, is an extremely complex phenomenon mediated by a large number of signaling cascades (24,25). The progression of metastasis involves cell migration from the primary tumor site, invasion of adjacent tissues, entry into and transport through the blood vascular system, reaching secondary sites, tumor growth and proliferation (26). Metastasis has been one of the most popular targets of anticancer studies, particularly for exploring therapeutic targets (27,28). Through the analysis of scutellarein-mediated suppression of cancer cell invasion and migration at the molecular level, the present study proved that scutellarein is a candidate compound for use in the prevention of cancer metastasis.

MMPs, including MMP-2, -9 and -14, which are overexpressed in tumor cells, aid migration and invasion by modifying the cellular microenvironment. Hence, small molecules or compounds inhibiting the expression of MMPs may prove to be beneficial to cancer therapy. However, several of the previously identified MMP inhibitors have failed in clinical trials, perhaps due to the large number of proteinases mediating enhanced tumor growth and progression (29). Therefore, the suppression of tumor growth is one of the critical factors in the treatment of cancer. Cancer cell growth and progression may occur due to inadequate apoptosis, which is initiated by extracellular receptor signaling and the proteolytic cascade (30). Accordingly, the induction of apoptosis in conjunction with the suppression of MMPs may be a potent mechanism for cancer treatment. In the present study, our results revealed that scutellarein not only decreased the expression of MMP-2, -9 and -14, but also induced apoptosis by suppressing the proliferation of HT1080 cells, thereby attenuating tumor development and metastasis.

The activation of NF-κB transcription factors is associated with several aspects of tumorigenesis, including cancer cell survival and proliferation, the prevention of apoptosis and an increase in the metastatic potential of tumor cells (31). Moreover, NF-κB expression in the nucleus contributes to the activation of MMP-2 and MMP-9, which play critical roles in cancer metastasis (32). Our results clearly demonstrated that the compound, scutellarein, potently inhibited the activation and nuclear translocation of NF-κB. Therefore, scutellarein may further decrease the expression of MMP-2, -9 and -14 through the NF-κB signaling pathway, thus inhibiting the migration and invasion of cancer cells.

In conclusion, scutellarein effectively suppressed the invasion and migration of HT1080 cells by inhibiting the expression and activity of MMP-2, -9 and -14, which are crucial enzymes in cancer metastasis. Scutellarein reduced cell proliferation by inducing the apoptosis of HT1080 cells. Furthermore, scutellarein suppressed tumor development in a nude mice injected with HT1080 cells, which demonstrated the stability and activity of scutellarein *in vivo*.

## Figures and Tables

**Figure 1:** Effects of scutellarein on viability of HT1080 cells. (A) Chemical structure of scutellarein (5,6,7,4′-tetrahydroxyflavone). (B) Toxicity of this compound on HT1080 cells, as determined by MTT assay (n=5). (C) Phase contrast images of the treated cells. HT1080 cells were treated with scutellarein (10 and 50 μm/l) or DMSO for 24 h. The values are the means ± SEM. ^**^P<0.01.

**Figure 2:** Scutellarein inhibits colony formation and induces the apoptosis of HT1080 cells. (A) Images of the cell colony assay showing stained colonies resulting from different treatments. (B) Quantification analysis of HT1080 cell colonies. (C) Effect of scutellarein treatment on the progression of the cell cycle in HT1080 cells analyzed by BD Cycletest assay. The values are the means ± SEM. ^**^P<0.01.

**Figure 3:** Scutellarein suppresses tumor growth in a mouse xenograft model. (A) Images of tumors removed from the mice in each group. (B) Weight (g) and (C) volume (cm^3^) of tumors separated from the treated mice. The values are the means ± SEM (n=6). ^**^P<0.01.

**Figure 4:** Scutellarein inhibits the migration and invasion of HT1080 cells. (A) Phase contrast images taken at the beginning (0 h) and after 6 h of the cell migration assay carried out using standard culture inserts. (B) The invasion of HT1080 cells was assessed using the Matrigel-coated Transwell system. The cancer cells were stained with crystal violet. (C) Quantification analysis of HT1080 cell invasion efficiency by measuring optical density at a wavelength of 600 nm. The values are the means ± SEM (n=3). ^**^P<0.01.

**Figure 5:** Effects of scutellarein treatment on the expression of matrix metalloproteinase (MMP)-2, -9 and -14. (A) mRNA expression of MMPs analyzed by RT-qPCR. The relative gene expression levels were calculated using the 2^−ΔΔCT^ analysis tool. Data are presented as the expression of MMPs compared to ACTB. (B) Representative zymographic analysis of MMP-2 and MMP-9 secreted by treated HT1080 cells. (C) Expression levels of MMPs in the treated cells analyzed by western bolt analysis. (D) Representative densitometric analysis of MMP expression by western blot analysis. β-actin and GAPDH were used as internal references in western blot analysis. The values are the means ± SEM (n=3). ^*^P<0.05, ^**^P<0.01.

**Figure 6:** Scutellarein inhibits the activation and nuclear translocation of nuclear factor (NF)-κB. (A) Western blot analysis of NF-κB signaling proteins in cytosolic and nuclear fractions. (B) Densitometric analysis of protein expression in the treated cells. β-actin and histone proteins were used as internal references for cytosolic and nuclear fractions, respectively. The values are the means ± SEM (n=3). ^*^P<0.05, ^**^P<0.01.

## Abbreviations

MMP: matrix metalloproteinase
NF-κB: nuclear factor κ-light-chain-enhancer of activated B cells
EMT: epithelial-mesenchymal transition
ECM: extracellular matrix
MTT: 3-(4,5- dimethylthiazol-2-yl)-2,5-diphenyltetrazolium bromide
DMEM: Dulbecco’s modified Eagle’s medium
DMSO: dimethyl sulfoxide
BSA: bovine serum albumin
FBS: fetal bovine serum
PBS: phosphate-buffered saline
RT-qPCR: quantitative reverse transcription- polymerase chain reaction
DEPC: diethyl pyrocarbonate
